The article "Traditional Chinese Medicine Recognition Based on Target Detection" was published in 2022. Journal: Evid Based Complement Alternat Med.

# Traditional Chinese Medicine Recognition Based on Target Detection

**DOI:** 10.1155/2022/9220443

**Published:** 2022-07-08

**Authors:** Bijun Lv, Liyao Wu, Tianran Huangfu, Jiaru He, Wenying Chen, Lu Tan

**Affiliations:** ^1^Department of Pharmacy, Yunfu Hospital of Traditional Chinese Medicine, Yunfu 527399, Guangdong, China; ^2^Department of Pharmacy, The Third Affiliated Hospital of Southern Medical University, Guangzhou 510000, Guangdong, China

## Abstract

Traditional Chinese medicine (TCM) is widely used in China, but the large variety can easily lead to difficulties in visual identification. This study aims to evaluate the availability of target detection models to identify TCMs. We have collected images of 100 common TCMs in pharmacies, and use three current mainstream target detection models: Faster RCNN, SSD, and YOLO v5 to train the TCM dataset. By comparing the metrics of the three models, the results show that the YOLO v5 model has obvious advantages in the recognition of a variety of TCM, the mean average accuracy of the YOLO v5 is 94.33% and the FPS has reached 75, this model has a smaller number of parameters and solves the problem of detection and occlusion for small targets. Our experiments prove that the target detection technology has broad application prospects in the detection of TCM.

## 1. Introduction

Traditional Chinese medicine (TCM) refers to prescription drugs that can be directly used in traditional Chinese medicine clinics or the production of preparations after processing Chinese herbs. It has a long history and is widely used in China. However, one of the dilemmas we face now is that there are too many varieties of TCMs in clinical use, even the same kind of TCMs may look different in appearance due to different production regions or processing and preparation techniques [1]. Some different types of TCM have small differences in appearance, making it hard to distinguish them from each other. At present, the dispensing of TCM is still largely dependent on the pharmacist manually [2], so misidentification of TCM is still unavoidable, even experienced pharmacists have difficulty in ensuring that no identification errors occur in their heavy workload. Medication errors caused by misidentification of TCM can affect the health of patients. As China's population continues to grow and age at an accelerating rate, it has brought about an increasing demand for TCM, while the traditional model of TCM personnel has a long cycle, and development is lagging behind the advancement of modern medical technology. Although the development of TCM is now strongly supported by the Chinese government, there is still a shortage of professionals in TCM. The continuous development of deep learning in recent years seems to bring opportunities for the development of TCM, with research in TCM diagnostic models [3,4], TCM toxicity component prediction [5], and TCM theory research [6], which also provides new methodologies for TCM modernization.

The article "Traditional Chinese Medicine Recognition Based on Target Detection" was published in 2022. Journal: Evid Based Complement Alternat Med.

In this article, we use the mainstream target detection algorithms represented by Faster RCNN, SSD, and YOLO v5 to train and test by constructing a TCM dataset in VOC format. Experiments show the potential of target detection technology to assist pharmacists with dispensing and verification. The main contributions of this study are the following:

- There are few attempts to introduce deep learning into TCM recognition, and this study explores the introduction of target detection into TCM recognition, which is a crossover study in the field of deep learning and TCM.
- There are few publicly available TCM image datasets, we have taken a large number of TCM images and completed manual labeling, and we will open up the datasets we have collected and labeled for evaluation testing in subsequent studies.
- This study compares different target detection algorithms applied to TCM recognition and analyzes the advantages and disadvantages of each, and the results show that YOLO v5 performs better than Faster RCNN and SSD. It provides a reference for subsequent studies.

## 2. Related Work

### 2.1. Literature Review

Previous studies of medicinal plants identification mainly focused on image classification by artificially set features. Herdiyeni [7], Mareta [8], and Song [9] classified medicinal plants images by extracting the variability in superficial features such as color, shape, or texture of medicinal plants by different classifiers. This kind of method could achieve satisfactory results, but as we mentioned above there are many types of TCM, so the manual setting of features is limited by the experience of the designer, the environment, and the location of the object, which leads to the lack of robustness of the features. In addition, the use of the manually setting features leads to a large computational effort of the model, and these deficiencies reduce the application scenarios and scope of the method Due to the continuous development of deep learning, Convolutional neural networks (CNN) have achieved outstanding results in computer vision classification and have been applied in many disciplines. CNN is characterized by the addition of convolutional layers and pooling layers; the new network structure can be formed based on different combinations and architectures of the convolutional layers and the pooling layers. In recent years, researchers have successively proposed a series of excellent deep learning models based on CNN, such as AlexNet (2012), VGGNet (2014), ResNet (2015), Inception (2015), DenseNet (2017), and so on, which have all performed well in various visual recognition competitions. For the first time, the AlexNet model [10] uses CNN for visual tasks in complex situations, replacing the Sigmoid function with the ReLu activation function, and preventing overfitting problems through dropout and image enhancement methods. VGGNet [11] and GoogleNet [12] improve the recognition accuracy of the model by continuously deepening the network structure, GoogleNet introduces the Inception module to reduce the number of parameters and increase the width of the model. By adding the residual module, ResNet [13] solves the problem that the error rate of the model does not decrease but increases when the number of network layers is greatly deepened and achieves a higher accuracy rate. DenseNet [14] is based on ResNet to connect all the layers with the dense connection, which reduces the number of parameters and makes the network more efficient. At present, some scholars have used CNN for the classification and recognition of Chinese medicine-related images. Huang et al. [15] proposed a network model that can be used to identify Chinese Herbal Medicine Leaves by improving the AlexNet model. Sun, et al. [16] used the VGG16 model to classify 95 Chinese herbal medicines with an average accuracy of 71%. The DenseNet-based recognition model proposed by Xing, et al. [17] could classify images of 80 Chinese herbal medicines with a maximum recognition rate of 97.3%. Liu, et al. [18] used GoogLeNet to classify images of 50 Chinese herbal medicine plants under complex background conditions, the accuracy of TOP-1 was 62.8%. In addition, a few studies used multiple models to compare results, Marwaha, et al. [19] used VGG16, MobileNet, Xception, and Inceptionv3 to classify the microscopic images of the two herbal plant powders with the highest accuracy of 96.4%. Azeez, et al. [20] compared the models of Inceptionv3, Resenet, MobileNet, and Inception-Resenet v2 to classify and identify 5 kinds of herbal plants, with an average accuracy rate of up to 95.5%. Tan, et al. [21] used different CNNs, including VGG, ResNet, Inceptionv4, and DenseNet to identify different types of Zanthoxyli Pericarpium. By comparing them with support vector machines and K-means clustering algorithms, the highest recognition accuracy of the CNN model is 99.35%, which is significantly higher than that of traditional detection and classification methods. Hu et al. [22] proposed to apply multitask learning to recognize Chinese herbal pieces pictures, and this study combined deep learning model and traditional features to improve model accuracy, and also achieved excellent results. Multitask learning enabled the model to have the ability to handle multiple tasks simultaneously, but for TCM recognition there seems to be no need to apply multitask learning, and as mentioned earlier, the manual design of features is laborious and relies on the designer's experience.

The article "Traditional Chinese Medicine Recognition Based on Target Detection" was published in 2022. Journal: Evid Based Complement Alternat Med.

From the research mentioned above, it can be seen that deep learning has shown excellent performance in the visual task of TCM detection, the current related research mainly focuses on the classification of TCM, that is, determining the category of the object based on the information in the image. Generally speaking, there are still many challenges and limitations in applying deep learning methods to the field of TCM image processing. For example, in the actual scene of TCM pharmacies, TCMs are often used in combination, which means that multiple TCMs are likely to be present at the same time. When the type and number of recognition targets are uncertain, if we want to know the specific location of the targets, the classification model alone is not enough to deal with the actual problem. Target detection requires identifying targets in an image and determining their location and class. Therefore, target detection is more practical than target classification in work, which provides a basis for the development of automated equipment to assist pharmacists.

Girshick et al. designed the RCNN based on CNN [23], which made a great improvement in the target detection efficiency of the model, and this technique has been developed rapidly on this basis. In recent years, many target detection models such as Faster RCNN, SSD, and YOLO have appeared in the field of target detection, and they have been widely used in many detection problems [24]. The current target detection algorithms are usually divided into two categories, a two-stage-detector represented by Faster RCNN and a one-stage-detector represented by SSD and YOLO. The advantages between the two are different: the two-stage-detector can achieve higher accuracy, but the generation of target candidate regions will slow down the speed; While the one-stage-detector can maintain a certain accuracy while not needing to generate target candidate regions first, the detection network can directly predict the object category and position, which has obvious advantages in detection speed. In previous studies, the application of a two-stage model or one-stage model transfer learning to the scope of TCM has mainly focused on TCM diagnosis [25,26], and there is no research on its application to image processing of TCM for the time being.

The article "Traditional Chinese Medicine Recognition Based on Target Detection" was published in 2022. Journal: Evid Based Complement Alternat Med.

The accuracy of the model is an important metric to determine whether the model can assist the pharmacist's work. Secondly, in a busy hospital scene, whether the model can complete real-time detection is not negligible. The calculation of the deep learning network model takes a lot of time to get the prediction results, and the role of the model in the daily work of the pharmacist is limited. Accurate identification of TCMs and rapid determination of their location are key technologies of the model. But we have not found any relevant research yet, so how to apply target detection technology to the work of pharmacists has research significance and potential application value.

### 2.2. Target Detection Algorithm

Faster RCNN [27] uses a region proposal network (RPN) instead of selective search, which saves the time required for detection and realizes target detection. The detection process is mainly after the image is feature extracted through the CNN, the RPN generates candidate regions of different sizes at each position of the extracted feature map, and finally, the Region Proposal is filtered by the Softmax function. The region of interest pooling is used to integrate the feature map of the CNN and the Region Proposal generated by the RPN, and then the classification is performed to confirm whether it is the detection target, and the position of the target is obtained through regression.

Liu et al. [28] proposed the Single Shot MulitBox Detector (SSD) target detection algorithm in 2016. SSD draws on the anchor mechanism of Faster RCNN and the end-to-end one-stage structure in which target classification and position regression are directly performed in convolution in the YOLO algorithm. The backbone network of the SSD algorithm is based on VGG16. The fully connected layers FC6 and FC7 are replaced with Conv6 and Conv7, the dropout layer and FC8 layer are removed, and adds some new convolutional layers for the extraction and prediction of multiscale feature maps. The advantage of multiscale is that feature maps of different sizes have different emphases on predicting objects. Large-scale feature maps generally contain more detailed information and focus on predicting small objects. Small-scale feature maps contain more global information and focus on predicting large objects.

Redmon et al. [29] proposed a regression-based target detection algorithm YOLO (You only look once) in 2016. YOLO provides a new idea for target detection, that is, using a simple structure of the convolutional network to directly complete the feature extraction, classification, and regression of target detection. YOLO divides the entire image into several grid cells, uses the center of each grid as the center of the bounding box to directly predict, and then eliminates bounding boxes with low probability through a threshold. This method significantly reduces the number of repeated calculations. Compared with the RCNN series of algorithms, YOLO has better overall performance. It realizes the end-to-end target detection process using a CNN, and the detection speed is faster. The YOLO series has been updated many times [30], and now it has launched the YOLO v5 version, which is an improved target detection network based on YOLO v4 [31] by Ultralytics LLC in 2020. The author's experimental results show that YOLO v5 [32] can greatly increase the speed of model calculations with almost no loss of accuracy, and provides an ONNX framework to convert between different models, which can be deployed to embedded and mobile phones. The main structure of YOLO v5 is similar to YOLO v4. As can be seen from Figure 1(a), YOLO v5 incorporates the Focus structure in the first layer of the backbone network. Suppose the input image size is 4 × 4 × 3, after slicing operation and channel concating operation, it becomes a 2 × 2 × 12 image, and then sends the 2 × 2 × 12 feature maps to convlutional layer to get the output. The Focus structure is added to transform the high-resolution image information from the spatial dimension to the channel dimension, which maximizes the preservation of the input information and reduces the input size, which is beneficial to improving the speed of training networks and inference.

The article "Traditional Chinese Medicine Recognition Based on Target Detection" was published in 2022. Journal: Evid Based Complement Alternat Med.

YOLO v5 references the Cross Stage Partial Network (CSPNet) in the backbone and neck sections, as shown in Figure 1(d) and 1(e), YOLO v5 uses two different CSP structures. The CSP structure with residual components is used in the backbone network for feature extraction, while the CSP structure in Neck uses convolutional operations instead of residual components. The CSP structure aims to divide the feature map into two parts, one part continues the convolution operation to obtain deeper feature information, and the other part is concated with the feature map after the convolution operation. The advantages of this design include: reducing computation, improving inference speed, reducing memory cost, and ensuring accuracy.

Spatial pyramid pooling (SPP) layer is added at the end of the backbone network due to the inconsistent size of the input images, which would increase the computation and consume a lot of training and inference time if reshape operation is performed on each image. The SPP layer, as shown in Figure 1(f), goes through different sizes of pooling layers to get the pooled output. The pooling kernel size and step size change adaptively according to the different image sizes during the maximum pooling, and the output of 1 + 4 + 16 dimensions is obtained after the SPP layer for any size of the feature map so that the size of the feature map input to the backbone network is no longer limited. In addition, the SPP layer plays an essential role in separating contextual features.

The article "Traditional Chinese Medicine Recognition Based on Target Detection" was published in 2022. Journal: Evid Based Complement Alternat Med.

In the Neck part of the network, YOLO v5 uses Feature Pyramid Network (FPN) and Path Aggregation Network (PANet). FPN is one of the more popular feature fusion methods that can be predicted separately on multiscale feature maps. The FPN algorithm is divided into two paths, one is bottom-top and the other is top-down, using a horizontal connection. Although the FPN structure adds less computation, this structure effectively fuses low-resolution, high-semantic feature maps with high-resolution, high-geometric feature maps. This enables the fused feature maps to have both high-level semantic features and low-level texture contour features, making full use of the features of different layers.

YOLO v5 takes reference from PANet and adds a bottom-top feature pyramid structure after the up-sampling of FPN for feature fusion. Different from PANet which uses the shortcut connection when fusing two feature maps, YOLO v5 fuses features by concating. After three different concating operations, three feature maps of different sizes are obtained, and then the CSP structure and convolution operations are added separately to make predictions on each of the three final feature maps.

The structure of FPN can extract strong semantic features from top-bottom, while the structure of PAN can extract strong positioning features from bottom-top. This method of fusing the feature maps of different layers of the convolutional neural network is more beneficial to feature extraction.

## 3. Methods

### 3.1. TCM Dataset

Since there is no public benchmark TCM dataset yet, we manually collected and labeled 2352 images, then expanded them to 23520 images by data augmentation, including Mirror flip, horizontal flip, rotation, contrast enhancement, affine transformation, mosaic enhancement, and divided the training set, validation set, and test set randomly according to the ratio of 6 : 2: 2.

The dataset covers 100 kinds of TCM images (shown in Figure 2). Considering the practical needs of the work, the dataset also includes some partially occluded, overlapping, multitarget and low-resolution images of TCM to fit the practical application scenarios to increase the robustness and generalization ability of the model. Unify the format of the dataset to the POSCAL VOC2007 format applicable to the three algorithms of Faster RCNN, SSD, and YOLO v5. We use the labelimg tool to mark the images, including the category and bounding box position information of the target to be recognized.

The article "Traditional Chinese Medicine Recognition Based on Target Detection" was published in 2022. Journal: Evid Based Complement Alternat Med.

### 3.2. Models Training

The experimental platform configuration of this article is computer operating system: Windows10, GPU: GeForce GTX 2080Ti, CPU: Intel(R) Core(TM) i7-10700, memory: Kingston 16G^*∗*^2 DDR4 3200Mhz. For the anchor selection, the anchor size of our dataset is obtained by k-means clustering instead of using the default anchor of the coco dataset. This approach allows the network to converge faster and learn the features of the images in our dataset better. The parameters that the network can learn to update include convolutional kernel parameters and bias parameters, but not Hyperparameter. Hyperparameters are manually set parameters that need to be specified before training and testing the network. Based on the experience of a large number of previous experiments, we analyzed and compared the optimal values of loss convergence, precision, and recall of the experimental results, and finally decided on the choice of hyperparameters. The initial learning rate of the weights is set to 0.001, and each batch contains 64 pictures. Momentum is set to 0.9, and the weight decay coefficient is set to 0.0001. The depth_multiple and width_multiple of the YOLO v5 model choose the default parameters, both of which are 1. The methods to avoid model overfitting in the experiments are as follows: 1) We randomly divide the dataset into training set, testing set, and validation set in the ratio of 6 : 2 : 2. In the process of training the model, the current constructed model is tested in each epoch using validation set to get the loss and accuracy. Comparing the accuracy of the validation set with the training set, If it performs well on the training set, but the performance on the validation set is bad, which indicates that the model is overfitting and we will stop training and analyze the cause, adjust the parameters and data, retrain the model. The experimental results show that our trained model performs well on the test set without overfitting. 2) When training the model iteratively, we set up an early stop mechanism to measure the performance of each iteration. When the validation loss starts to increase, the training of the model is stopped to prevent overfitting. 3) We increase the number of training samples through data augmentation, including horizontal flip, affine transformation, Mosaic data augment, etc. Using dropout to increase regularization in training the model can also prevent overfitting.

### 3.3. Evaluation Metrics

There are some important algorithm evaluation metrics in target detection including precision, recall, mean average accuracy (mAP). It is defined as follows:

(1) $$\begin{array}{c} \text{Precision}=\frac{T_{P}}{F_{P}+T_{P}}, \end{array}$$

(2) $$\begin{array}{c} \text{Recall}=\frac{T_{p}}{F_{p}+F_{N}}, \end{array}$$

(3) $$\begin{array}{c} AP=\int_{0}^{1}p\left(r\right)dr, \end{array}$$

(4) $$\begin{array}{c} mAP=\frac{1}{n}\sum_{i=1}^{n}APi. \end{array}$$

In the formula, True Positive (*T*_*P*_) is judged as a positive sample and it is a positive sample in fact; False Positive (*F*_*P*_) is judged as a positive sample and it is a negative sample in fact; False Negative (*F*_*N*_) is judged as a negative sample and it is a positive sample. Average accuracy (AP) is the average accuracy for a certain category, mAP is the mean average accuracy of all categories.

The article "Traditional Chinese Medicine Recognition Based on Target Detection" was published in 2022. Journal: Evid Based Complement Alternat Med.

## 4. Results and Discussion

### 4.1. Results for Different Epochs

The experiment recorded the values of Precision, Recall, and mAP of the three models at different Epochs. It can be seen in Figure 3 that, with the increase of Epochs, the metrics of the three models are also increasing, which means that the detection effect of the network model is better. After 45 Epochs, YOLO v5 performed better than Faster RCNN and SSD for the same Epochs.

### 4.2. The Results of Evaluation Metric

The comparison results of the three models on the TCM test set are shown in Table 1. Compared with Faster RCNN and SSD, the precision of the YOLO v5 model has increased by 11.15% and 17.86%, the recall has increased by 8.40% and 15.53%, and the mAP has increased by 8.77% and 13.01%, respectively. The results of these metrics showed that the YOLO v5 model outperformed both the Faster RCNN and SSD on the same TCM dataset. Our experimental results are similar to those of other studies that have applied target detection to medical images. For example, Zhao et al. [33] proposed the use of YOLO v5 and SSD for the real-time detection of blood cells. The authors trained and validated two target detection networks using a blood cell dataset that included red blood cells, white blood cells, and platelets. The experimental results showed that the mAP of YOLO v5 was 0.96, while the mAP of SSD was only 0.62. In terms of detection speed, the detection frame rate of YOLO v5 can reach 62 FPS, which is almost 100 times that of SSD. This demonstrated that YOLO v5 was more accurate in identifying blood cells and could detect them in real-time, making it more suitable for clinical applications than SSD. Qu et al. [34] applied YOLO v5 and Faster RCNN to the CT image detection of COVID-19 and conducted a comparative experiment using the same dataset. The results showed that the mAP of YOLO v5 reached 0.623, while that of Faster RCNN was only 0.466. YOLO v5 showed significant advantages in identifying and localizing COVID-19 abnormalities on chest radiographs, providing greater practical value in clinical practice.

The article "Traditional Chinese Medicine Recognition Based on Target Detection" was published in 2022. Journal: Evid Based Complement Alternat Med.

### 4.3. Real-Time Comparison of Models

The common metric for evaluating the detection speed of the model is Frames Per Second (FPS). The FPS of the three models under the same experimental setting is shown in Figure 4. YOLO v5 can detect 75 images per second, and the detection speed is more than 58% higher than that of SSD. And two-stage detector Faster RCNN of the FPS is only 4, significantly behind in comparison with the other two models, it is difficult to achieve real-time recognition, which limits its potential applications. The FPS of the YOLO v5 and SSD models in this experiment has reached the effect of real-time detection, which proves that the one-stage algorithm has more advantageous than the two-stage in terms of detection speed. The SSD algorithm outputs candidate regions for each convolutional layer during the operation, resulting in more candidate regions generated than YOLO v5, so the detection speed is slow.

### 4.4. Parameter Size Comparison

The model can be deployed through the front-end to avoid network latency in data propagation, but running the model requires loading weights, and a large number of parameters will occupy the running memory of the device resulting in slower operation, and the size of the model parameters affects the deployment cost of the device. Although the model size can be reduced by model compression, this method tends to reduce the accuracy of the model, so it is more appropriate to choose a model with a smaller number of parameters while ensuring accuracy and real-time performance. The parameter sizes of the three network models are shown in Figure 5, the parameters of YOLO v5 are significantly smaller compared to the other two models. The CSP module of YOLO v5 can optimize repeated gradient information through the use of split and merge strategies across stages, and effectively reduce model parameters. Therefore, the deployment cost of YOLO v5 is lower, and it is easy to quickly deploy and upgrade online.

### 4.5. Results of Actual Sample Tests

In order to visualize the recognition effect of Faster RCNN, SSD and YOLO v5 on TCM mentioned in this paper, we randomly selected samples from the test dataset in the three algorithms for comparison. As shown in Figure 6, the YOLO v5 network can detect the missed targets of Faster RCNN and SSD, which is more advantageous in dealing with the problems of small target detection and target occlusion, and can complete the detection task well in practical scenarios. This may be related to Mosaic Augmentation, which allows random scaling, distribution, and stitching of images to produce more data and improve the accuracy of the YOLO model for small target detection.

The article "Traditional Chinese Medicine Recognition Based on Target Detection" was published in 2022. Journal: Evid Based Complement Alternat Med.

## 5. Conclusion and Future Work

In this article, we briefly introduce the development of CNNs and target detection algorithms, focusing on the comparison of three current mainstream target detection methods, namely Faster RCNN, SSD, and YOLO v5, and then train and test the three models using TCM datasets. It is concluded that the recently released YOLO v5 model has significant advantages over faster RCNN and SSD in terms of mAP, FPS, parameter size, and actual detection effect of target detection for TCM.

Overall, the deep learning-based target detection algorithm provides a new way of thinking and approach for TCM detection, not only to identify specific targets in images, but also to determine where the targets are located, with the advantages of accuracy, speed, and ease of deployment. The target detection model can effectively reduce labor input and reduce the work intensity of pharmacists by performing operations related to detection of TCM in specific scenarios, and the application prospect is wide. Through the analysis of the experimental results, we found the direction of model performance improvement. In further work, we will try to reduce the time required for model inference through model pruning and lightweight with almost no loss of accuracy, so that the algorithm is suitable for TCM detection in real scenes. In addition, we will continue to supplement the dataset to ensure the comprehensiveness of the TCM dataset.

## Figures and Tables

**Figure 1:** YOLO v5 network structure diagram.

**Figure 2:** Example images of TCM.

**Figure 3:** Relationship of epochs with mAP, precision, and recall.

**Figure 4:** FPS of deep learning models.

**Figure 5:** Parameter size of deep learning models.

**Figure 6:** The detection results of test images. (a) the detection result of the image in the Faster RCNN; (b) the detection result of the image in the SSD; (c) the detection result of the image in the YOLO v5.

**Table 1:** Evaluation of deep learning models.

Algorithm	Precision/%	Recall/%	mAP/%
Faster RCNN	85.12	86.71	85.56
SSD	78.41	79.58	81.32
YOLO v5	96.27	95.11	94.33

## Data Availability

The data used to support the findings of this study are available from the corresponding author upon reasonable request.
